This article has been retracted.

# Application of Mathematical Model Using Random Forest in Performance Appraisal Management of Cadres in Free Trade Zone

**DOI:** 10.1155/2022/6964582

**Published:** 2022-08-12

**Authors:** Jie Zhang

**Affiliations:** Department of Business Administration, Chaohu University, Hefei 238024, China

## Abstract

To improve the efficiency of scientific assessment of cadre performance, first, this work analyzes the current situation of cadre performance appraisal in the free trade zone under the background of big data, and introduces the free trade zone and Random Forest (RF) algorithm. Second, based on the cadre evaluation index, this work establishes the cadre performance evaluation system of the free trade zone. Finally, the random forest algorithm model is implemented for the performance evaluation of cadres in the free trade zone. Additionally, the model's performance is verified with the actual data, including the acquisition of the best parameters and the most important indicators of the model and the performance comparison between the RF algorithm and other models. The results show that the performance of cadres in the free trade zone is finally divided into four grades: medium, good, qualified, and excellent. There are obvious grade differences in the performance of cadres in the free trade zone. Partly because some qualified cadres lack a strong sense of competition and professional competence, do not publicize the work of cadres in the free trade zone, and do not communicate with the masses in time. In the data processing, 18 missing experimental data were supplemented, and the best model parameters were obtained as follows: NTree = 200, MTry = 1. The most important indicators of cadre performance evaluation are the construction of a clean and honest government, the ability to act in accordance with the law and the professional ability. The accuracy of the RF algorithm obtained here is 71.4%. The prediction accuracy of the RF algorithm for the overall sample, training sample, and test sample is 94%, 96%, and 86%, respectively, which are higher than those of other common models. A RF algorithm with good classification effect is obtained and this work provides a reference for the scientific management of cadre performance appraisal.

## 1. Introduction

Scientific cadre performance appraisal plays a very important role in cadre work, which is the motivation of this work. With the arrival of China's social and economic transformation, under the new normal of political economy, party and government cadres at all levels are faced with a new issue of how to transform government agencies from market managers to market service providers, thus better serving the main body of the market economy [1]. In the process of this transformation, the performance appraisal of government cadres has played a huge role. The performance assessment adopts scientific methods to assess the work objectives and performance standards of party and government cadres, and evaluate their work completion and performance [2]. With the continuous development of big data technology, governments at all levels have introduced more scientific assessment methods for the performance assessment of party and government cadres, including policies, terms, laws, and regulations, which provide standards and basis for the performance assessment of party and government cadres. The western developed countries have used the enterprise management model for reference and introduced the market competition mechanism to improve the administrative efficiency of the examinees. China's current administrative assessment has drawn on foreign advanced experience. Some scholars have made a comprehensive analysis of the performance appraisal measures implemented in China from a legal perspective, including the legislative background of the civil servant law, and conducted an in-depth and detailed analysis of the civil servant law [3].

The free trade zone is where the member states of the free trade agreement completely cancel the tariffs and quantitative restrictions on commodity trade for the free flow of commodities among the member states [4]. Under the background of the new normalization of politics and economy, higher requirements are put forward for the government management functions of Party and government cadres in the free trade zone. The government management system can keep up with economic and social development only by continuously optimizing the care performance appraisal system and promoting the construction of leading cadres [5, 6]. The era of big data has come. It has become urgent to optimize cadre performance appraisal systems through new technologies in the free trade zone under scientific and reasonable planning. One method, in particular, is the random forest (RF) algorithm, which is widely used in many fields, such as economics and management with its excellent classification ability and prediction accuracy [7, 8].

At present, the cadre performance appraisal lacks scientificity and objectivity. Based on the RF algorithm, this work proposes a mathematical model for the performance appraisal management of cadres in the free trade zone. It provides a more scientific and comprehensive appraisal scheme for the performance appraisal of cadres in the free trade zone. This work introduces the current situation of cadre performance appraisal, and summarizes the problems existing in cadre performance appraisal. Moreover, this work introduces the RF algorithm, establishes the cadre performance appraisal system, realizes the RF algorithm model of cadre performance appraisal, and carries out empirical research on this basis. The research innovatively applies RF algorithm to the performance appraisal of cadres in the free trade zone, thereby improving the scientificity of the performance appraisal of cadres. This work provides a positive reference for establishing a scientific assessment system for leading cadres in the free trade zone.

## 2. Research Status of Cadre Performance Appraisal

Internationally, the research on government performance appraisal has begun as early as the 18th century. The performance appraisal of leading cadres is inspired by the theories of enterprise human resource management and draws lessons from enterprise efficiency models and methods [9]. Since the 20th century, the focus of international research on government performance has been on internal appraisal. That is, the performance appraisal of cadres is based on criteria, such as management ability, management efficiency, public satisfaction, and service quality [10]. While the 21st century is witnessing the center of performance appraisal of government cadres shifting towards the importance of people in the organization, which pursues the dynamic balance between people and decision-making [11]. After years of exploration, the new public management theory is put forward, which further deepens the previous research, introduces the market competition mechanism into the appraisal system, and provides new standards for the reform of government work [12, 13].

Domestically, several definitions of performance prevail. (1) Performance is the result. (2) Performance is behavior. (3) Performance is the quality of employees [14]. The research on government performance appraisal in China has a late start. Not until the end of the 20th century, China realizes the improvement of administrative efficiency in government management [15]. After years of development, domestic government management performance appraisal has been transformed from internal work to external work, which is in line with result-oriented international standards [16]. Relatively, the research on the performance appraisal of civil servants in China has started earlier, with a mature system, which is mainly studied from the legal perspective [17]. Many foreign performance appraisal experiences are referred to in the research on performance appraisal of the domestic government department, combined with China's national conditions, thus forming a government performance appraisal index system with Chinese characteristics [18]. The research on the performance appraisal system indicates that the subjective indexes have a great impact on the domestic performance appraisal, the accuracy of the performance appraisal results is low, and the appraisal results cannot truly reflect the work performance of Party and government cadres [19].

In order to meet the scientific principle of performance appraisal, many places have tried the form of third-party evaluation of government performance according to the local actual situation. Many scholars have also done a lot of research on local government performance appraisal. Although China has made fruitful achievements in cadre performance appraisal in recent years, compared with western developed countries, the current cadre performance appraisal system is still immature and has some shortcomings. There is still much room for improvement from the overall analysis of the research. At present, most studies are mainly confirmatory and lack exploratory research. To improve the effectiveness of our government performance appraisal, it is necessary to strengthen the exploratory research, which should focus on quantitative analysis and empirical research. Currently, there are still some problems in the research, such as too simple assessment indicators, not obvious incentive effect of performance assessment, and the asymmetry of assessment information between the assessor and the assessed. Therefore, the RF algorithm is creatively introduced into the cadre performance appraisal to achieve a more accurate and scientific performance appraisal model.

## 3. Implementation of Cadre Performance Appraisal System and RF Model in the Free Trade Zone

Here, the performance appraisal system of cadres in the free trade zone is constructed through specific analysis. Notably, the performance appraisal of cadres in the free trade zone differs from that of leading cadres in other regions by highlighting the work indexes with free trade economic characteristics, such as innovation in political management and the promotion of free competition and market opening of enterprises. Meanwhile, the performance appraisal of cadres in the free trade zone underlines the transparency of appraisal information, accepts public supervision, and prioritizes the legal system construction and relevant indexes. Particularly, Handling affairs according to the law has become an important appraisal index in the performance appraisal for Party and government cadres [20].

The objectives of performance appraisal of cadres in the free trade zone include efficiency, fairness, economy, and effectiveness. The general framework of performance evaluation indexes for cadres in the free trade zone is shown in Figure 1.

Figure 1 illustrates that there are three indexes: the performance, work cost, and management effect of Party and government cadres in the free trade zone. The indexes are composed of three levels: comprehensive evaluation indexes as the target level, classification evaluation indexes as the factor level, and single evaluation indicators as the sub-index level. Thereupon, the comprehensive performance indexes of cadres in the free trade zone should include legal construction indexes, economic development indexes, social development indexes, ecological environment indexes, people's life indexes, public satisfaction indexes, and characteristic indexes of the free trade zone.

The specific appraisal contents of each index are the work results of town and street leading cadres and leading cadres of district authorities, as detailed in Table 1.

Table 1 presents that the performance appraisal indexes of cadres in the free trade zone cover 6 categories, each of which contains 19 different single indexes. Shen and Ho proposed a large-scale data research method based on cluster analysis [21]. Here, the K-means clustering algorithm is adopted for the classification standard of cadre performance appraisal in the free trade zone, which can effectively process data and classify samples according to the category of fewer sample data, with high classification accuracy. K-means clustering algorithm generates K data subsets by processing the given data and then divides them into C categories. The clustering goal is to obtain the data set with the minimum sum of squares [22]. The category center in each category is the judgment standard of distance. Equation (1) shows the calculation method of the sum of squares of distances of each distance center.

(1) $$\begin{array}{c} Q\left(f_{k}\right)=\sum_{x_{1}\in f_{k}}{\left\|x_{1}-P_{k}\right\|}^{2}. \end{array}$$

In equation (1), *Q* represents the sum of squares of the distance center, *f*_*k*_ denotes the classification, *x* indicates the data set, and *P*_*k*_ is the distance center.

(2) $$\begin{array}{c} Q\left(F\right)=\sum_{k=1}^{k}Q\left(f_{k}\right)=\sum_{k=1}^{k}\sum_{x_{1}\in f_{k}}{\left\|x_{1}-P_{k}\right\|}^{2}. \end{array}$$

In equation (2), F represents the sum of the divided categories. K-means clustering algorithm initializes the data set, groups, determines the classification center, and repeats the steps of grouping and determining the center until the algorithm converges.

Here, the performance data of cadres in the free trade zone are collected from the government platform of the study area. Totally, 110 pieces of data are collected, of which 18 are missing. Afterward, the missing data are removed, and the K-means clustering algorithm is used to cluster the complete 92 pieces of data, and the clustering results are based on the smallest class.

## 4. Implementation of RF Model for Cadre Performance Appraisal Management in the Free Trade Zone

### 4.1. Principle of RF Model

RF model is an algorithm with higher prediction accuracy evolved from a single decision tree algorithm. RF algorithm randomizes variables and training samples. When the new sample is input into the RF model, each decision tree in the forest will classify the sample. RF algorithm introduces randomness into the model, reduces the correlation between decision trees, and improves the prediction accuracy of the algorithm while ensuring the accuracy of each decision tree [23]. The construction process of RF is shown in Figure 2.

Figure 2 reveals that the core of the process of RF algorithm is sample randomization, RF decision-making, and decision tree result classification. Each decision tree in the RF is a binary tree, which splits recursively from top to bottom. The training data are stored in the root node of the binary tree. According to the principle of minimum node purity, the root node does not stop splitting until the termination condition of branching is met. The input preparation of the RF algorithm is very simple. The diversified subtree structure of the RF algorithm can process massive amounts of data more efficiently. Compared with other traditional algorithms, the RF algorithm is advantageous in time-consuming.

The software tools used in this work are open source software R language and Matlab software. The “random Forest” package in R software can easily establish RF models. Because R language has stronger object-oriented function than other programming languages, the software is widely used, including Google and Facebook. The data processing flow of the RF algorithm is shown in Figure 3.

Figure 3 shows the detailed processing steps of the data set in the RF algorithm, and the regression and classification of the predicted value output by the RF algorithm are expressed as in equations (3) and (4).

(3) $$\begin{array}{c} f\left(x_{t}\right)=1\frac{1}{N_{\text{tree}}}\sum_{t=1}^{N_{\text{tree}}}s_{t}\left(x_{t}\right), \end{array}$$

(4) $$\begin{array}{c} f\left(x_{t}\right)=\text{majority vote}\left\{s_{t}\left(x_{t}\right)\right\}\begin{array}{c} N_{\text{tree}}\\ t=1 \end{array}. \end{array}$$

Equation (3) is the regression equation of the RF algorithm, where *s*_*t*_ and *x* represents the decision tree and the sample to be tested, respectively. Equation (4) is the classification equation of the RF algorithm.

In the RF algorithm, different training sets are generated by the bagging method. The random feature selection is used to generate the new training set to obtain the decision tree and prune the decision tree [24]. The new training set has been sampled by bootstrap, but part of the training set obtained by the bagging method will not appear in bootstrap samples, which is called out of bag data, and the estimation model implemented by out of bag data is called out of bag data estimation [25]. The relevance of the decision tree in the RF algorithm is reduced mainly by the linear combination of a random selection of feature variables [26].

### 4.2. Implementation of RF Model for Cadre Performance Appraisal Management in the Free Trade Zone

Here, the original data set comes from the government official website, National Statistics website, and social networks. The data types are complex and the data sources are wide, which happens to be the characteristics of big data. The collected data include statistical data on the promotion of key projects of cadres in the free trade zone, as well as mass satisfaction feedback. Finally, 110 pieces of data are collected, with 18 missing and 92 complete.

Firstly, the collected data are preprocessed, and the missing data are supplemented to lay the foundation of performance appraisal with a complete set of data. Specifically, the missing data are supplemented through the Expectation-Maximum (EM) algorithm with efficient iteration, and the EM algorithm can perform maximum likelihood estimation for missing data [27]. The EM algorithm iteratively processes the continuous data conforming to the normal distribution and maximizes the missing data. The specific calculation reads:

(5) $$\begin{array}{c} Q\left(\theta |\theta^{\left(t\right)}\right)=E\left\{\log\;f_{Y}\left(y|\theta \right)|x,\theta^{\left(t\right)}\right\}. \end{array}$$

In equation (5), *θ* represents the missing data, *θ*(*t*) indicates the maximum point under t-times iteration, *Q* denotes the joint log-likelihood expectation, and *E* stands for the expectation. The obtained results are tested for normal distribution. When the test results conform to the normal distribution, the EM algorithm can be used to supplement the missing data. Firstly, the EM algorithm is used to estimate the parameters of missing data, then the mode is used to supplement the discrete data and retrograde data, while the *E* value and *M* value determined in the EM algorithm are used to supplement the continuous data, and thus the supplementary data are classified [28].

The open-source software R language with random Forest package is adopted to implement the RF model for the performance appraisal of cadres in the free trade zone. The object-oriented R language has been widely used in data analysis. The main functions of the R language used in the proposed model include random Forest function, Importance function for listing important factors, vary plot function for drawing important factors, and Predict function for model prediction.

The experimental data sample is small in scale. First, the sample size is expanded, and pseudo data are introduced. The research shows that when the pseudo data size reaches 200, the predictability of the RF model peaks [29], and 30% of the data are used to measure the predictability of the model, while 70% are used to build the training sample model. RF algorithm is not sensitive to the unit and dimension of data, so data normalization is not needed.

Parameters of RF include MTry, XText, and NTree. NTree represents the number of decision trees in the RF model, and the larger the NTree is, the better the classification effect of the RF model is, but the slower the processing speed of the model will be. Therefore, there is an optimal number of trees in the model. Previous studies have shown that the optimum NTree is 200 and 300. Accordingly, the experimental analysis is conducted to obtain the optimum NTree. MTry indicates the number of selected eigenvalues at the nodes in the RF model. Here, 19 eigenvalues are selected, so initially Mtry = 19. Meanwhile, NTree and MTry values of the model are tested. The performance of the model is characterized by the error rate of the model. The error rate of out-of-bag data can evaluate the importance of appraisal indexes and is directly affected by the change of the number of indexes in the RF model. Thus, the error rate of out-of-bag data can be used to evaluate the performance of the model. Further, based on the error rate of out-of-bag data, the importance of the above 19 indexes is scored on a 5-point system, The scoring results are tested and obtained from the training data set in the R language package. That is, the training data set and random Forest and VarSelRF are chosen from the R language package for the experimental data set and program packages. The importance measurement of each index is given later. Finally, seven pieces of data samples of cadres' performance appraisal in the free trade zone are selected to evaluate the predictability of the RF model. The characterization method is realized by comparing the predicted value of the model with the real value. (1) means excellent, (2) represents good, (3) indicates medium, and (4) suggests qualified. Next, the model accuracy of the RF model is compared with other models under the distribution of three quantitative proportions of data sets, which are the regression tree classification model and the Bayesian network model. The comparison of the number of samples between the training set and test set in the three quantitative proportions is 1 : 1, 3 : 2, and 3 : 3, respectively. The evaluation results are given in the following section.

## 5. Analysis Results of RF Algorithm Model for Cadre Performance Appraisal in the Free Trade Zone

### 5.1. Analysis of Data Set Clustering Results

The best results obtained by the K-means clustering algorithm are shown in Table 2.

Table 2 displays that the best results obtained by the K-means clustering algorithm are four categories, that is, when the performance appraisal results of cadres in the free trade zone are four categories, the overall error is the smallest. Meanwhile, the fourth type of cluster data accounts for the highest proportion, up to 35.9%, the first type of cluster data accounts for 23.9%, the second type of cluster data accounts for 19.6%, and the third type of cluster data accounts for 20.7% of the total data amount. Previous studies imply that the proportion of clustering data is related to data classification. In the cadre performance appraisal, the proportional distribution of data at different levels presents a certain state, that is, the proportion of data with medium results in the cadre performance appraisal is the highest, the proportion of data with good results is the second, and the proportion of data with qualified and excellent results is the smallest. Therefore, combined with Table 2 and previous studies, the performance appraisal standards of cadres in the free trade zone are classified into four categories: medium, good, qualified, and excellent.

Under the comparison of the excellent data and qualified data in the performance appraisal of cadres in the free trade zone, the differences between the two types of data are mainly in three aspects: the executive power of cadres in the free trade zone, the standardization in work, and the satisfaction of the masses. This is because the performance appraisal results of qualified cadres in the free trade zone do not have a strong sense of competition, the professional level for some important work is not high, the publicity of the work of cadres in the free trade zone is not enough, and the communication with the masses in the process of work is not timely.

### 5.2. Analysis of Data Fitting Results

In the data preprocessing of the RF algorithm, the normal distribution test results of continuous data from some samples are shown in Figure 4.

Figure 4(a) demonstrates that the distribution results of the data roughly obey the normal distribution, and the errors at both ends of the distribution curve are large, which may be due to a large number of economic development statistics in some government units. Similarly, Figure 4(b) displays that the data distribution results obey the normal distribution. Therefore, based on the previous sections and the EM algorithm, the missing data are supplemented. There are 18 pieces of missing data in this experiment, all of which are supplemented.

### 5.3. Experimental Results of Optimal Parameters

The experimental results of the optimal parameters based on the model error rate are shown in Figure 5.

Figure 5 shows that when NTree is equal to 200 or 300, the error rate of RF model increases with the increase of MTry value. When MTry = 19, both curves reach the maximum value, exceeding 50%. In general, the model error rate when NTree = 200 is lower than that when NTree = 300. When MTry = 1, the error rate of the model is the smallest. Therefore, the best model parameters selected here are NTree = 200 and MTry = 1.

### 5.4. Measurement Results of Index Importance

The scores of the performance appraisal indexes of cadres in the free trade zone are shown in Table 3.

Table 3 suggest that the most important performance appraisal indexes of cadres in the free trade zone are the Construction of Party style and clean government, Handling affairs according to law, and Professional Competency, which is consistent with China's focus on cadre performance appraisal in recent years, paying more attention to cadres' ability to handle affairs according to law and self-management, and the importance of leadership and innovation ability is also high. Here, the research is conducted on a free trade zone, and the performance appraisal of cadres in this region has high requirements for innovation ability. In this appraisal index system, the work related to employment and the ecological environment is promoted by professionals, so the importance of expanding employment and the ecological environment is relatively small.

### 5.5. Evaluation of Model Predictability

The comparison between the prediction of the proposed model and the true results under seven sets of sample data is shown in Figure 6.

Figure 6 shows that the accuracy of the proposed RF model is high. The prediction of samples 1, 2, 5, 6, and 7 are consistent with the true results. The prediction grade of sample 3 is good, while the true grade is medium, and the prediction grade of sample 4 is medium, and the true grade is good. Hence, for the seven samples selected, the accuracy of the proposed RF model is 71.4%, indicating that the predictability of the model is good.

Further, the comparison results of prediction accuracy of different models are shown in Figure 7.

Figure 7 shows that the proposed RF model for cadre performance assessment in the free trade zone has high prediction accuracy. The prediction accuracy of the whole sample is 94%, and the overall error rate is 6%. The prediction accuracy of training samples is 96%, and that of test samples is 86%. The prediction accuracy of Bayesian network model is slightly lower than that of RF model. The prediction accuracy of three groups of samples is 89%, 92%, and 77%, respectively. The prediction accuracy of regression tree classification model is the lowest, the overall sample accuracy is 53%, the training sample accuracy is 47%, and the test sample accuracy is 77%. Obviously, the accuracy of the proposed RF model is higher than that of the regression tree model and Bayesian network model, and the accuracy of the training samples is higher than that of the test samples as a whole. This indicates that the model does not have over-learning, and the classification results are generally good. The results show that the proposed RF model has good classification effect and is feasible in general.

## 6. Conclusions

Based on improving the objectivity and scientificity of the current cadre performance appraisal, this work studies the RF algorithm. This work introduces the background of cadre performance appraisal, and comprehensively analyzes the performance data of cadres in the free trade zone from the aspects of mass satisfaction, quality, performance, and expected efficiency in accordance with the specified standards and the established appraisal system in combination with mathematical statistics and operational research principles. Finally, it is found that the prediction accuracy of this model is high, and the prediction accuracy of the whole sample is 94%, which is higher than that of other models. The most important performance evaluation indicators for cadres in the free trade zone are the construction of a clean and honest government, handling affairs according to law and professional competence. This work provides a reference for the performance appraisal management of cadres in the free trade zone under the big data. Whereas there are still some shortcomings. The data set collected in this work is limited, so the research coverage is very small, and the determination of indicators and the construction of indicator system also need to be further optimized. The research on the application of random forest algorithm in cadre performance appraisal is not deep enough. Therefore, the future work will increase the number of data sets, add more research indicators, and deeply analyze the application status of the RF algorithm in cadre performance appraisal, to conduct more in-depth research and finally optimize the research results.

## Figures and Tables

**Figure 1:** General framework of performance evaluation indexes for cadres in the free trade zone.

**Figure 2:** Implementation of RF algorithm.

**Figure 3:** Data processing process of RF algorithm.

**Figure 4:** Data distribution results. (a) represents the distribution result of the “economic development” data set, and (b) indicates the distribution result of the “people's living standards” data set.

**Figure 5:** Analysis results of optimal parameters.

**Figure 6:** Comparison between prediction grade and true grade of the RF model.

**Figure 7:** Comparison of prediction accuracy of different models.

**Table 1:** Performance evaluation indexes of cadres in the free trade zone.

Classification index	Single index
Ability to perform duties	Economic development, people's living standards, social development, and ecological environment

Key work of the free trade zone	The key work of each district, street, and town unit around the central work

Routine work	Routine work carried out by district and street units

Mass satisfaction	Act per the law, make pragmatic innovations, make scientific innovations, build grass-roots democratic politics, comprehensively manage social security, expand employment and social security, manage primary and secondary education, and improve the production and living environment

Leading cadres' self-test indexes	Leadership, construction of party style and clean government, and ideological and political construction

Evaluation index of moral and talent quality of leading cadres	Professional competency and policy level

**Table 2:** Data set clustering result distribution.

Classification	Data proportion (%)
Cluster 0	23.9
Cluster 1	19.6
Cluster 2	20.7
Cluster 3	35.9

**Table 3:** Index importance scores.

Index serial number	Fractional value
Economic development	3.2
People's living standards	3.4
Social development	2.2
Ecological environment	1.4
The key work of each district, street, and town unit around the central work	3.8
Routine work carried out by district and street units	2.8
Handling affairs according to law	4.3
Pragmatic innovation	3.5
Scientific innovation	3.9
Grassroots democratic political construction	2.9
Maintain public security in a comprehensive way	2.7
Expand employment and social security	1.4
Primary and secondary education management	1.8
Improve production and living environment	2.5
Leadership	3.9
Construction of party style and clean government	4.5
Professional competency	4.2
Political and ideological construction	3.7
Policy level	2.9

## Data Availability

The data used to support the findings of this study are included within the article.
